The article "University Network and New Media Advertising Teaching Design Features and Influence: Environmental Perspective Analysis in Campus Humanistic Governance" was retracted in 2023. Reasons: signs of a paper mill; suspected computer-generated content; unreliable results or conclusions; concerns about the data.

# University Network and New Media Advertising Teaching Design Features and Influence: Environmental Perspective Analysis in Campus Humanistic Governance

**DOI:** 10.1155/2022/6380719

**Published:** 2022-07-21

**Authors:** Jing Zhang

**Affiliations:** Department of Literature, Modern College, Northwest University, Xi'an 710130, China

## Abstract

Under the background of network development in the new era, the integration of multimedia technology and information technology promotes the development of teaching environment. Based on the influence of humanistic governance environment, the university network environment and the advertising teaching environment are constantly integrating new elements with the development of the times, becoming the key point to guarantee the teaching quality. In the research, the relevant data and information were collected and analyzed by the methods of inference and induction analysis. According to the sensory parameters of students' cognitive emotions (*n* = 64, *a* > 0.847), the standard deviation was 0.810/0.695 and the action was 0.927/0.655. How to construct the university network and advertising teaching environment were explored. And, in view of the design of the environment characteristics as well as the impact on students, the purpose was to ensure that students had a good learning environment, which could improve the learning efficiency.

## 1. Introduction

At present, a good learning adaptability is an inevitable requirement to improve the quality of talent training in the era of knowledge economy. Under the influence of campus humanistic governance environment, the teaching environment design of university network and new media advertising has a direct impact on students' learning quality. In the past, students had problems of maladaptation in the process of learning and the influence of learning environment on students led to the lack of adaptability [1]. As for the existing problems, designing a quality environment mobilizing students' self-efficacy in learning has a direct and significant impact on learning adaptability. Three rounds of teaching practice were carried out to verify the effect of the intervention model from two aspects of students' procedural performance and result-oriented performance. According to the implementation effect of each round, the intervention model and its application were reconsidered and improved to gradually improve the learning adaptability of university students [2]. In the environment governed by humanities colleges and universities, the use of advanced network and new media teaching has a positive impact and importance on reducing the pollution and carbon emissions produced by the traditional teaching process. Therefore, adopting advanced network teaching means is conducive to environmental protection. On the other hand, taking the methods of new media–related technology can create an environment of clean and green space.

As the representatives of the emerging technology, Mobile Internet, cloud computing, and virtual reality technology present a blowout development, which reconstructed social economy, cultural life, and other aspects. They are integrated in all walks of life rapidly, so that more ordinary consumers can also deeply participate in the process of scientific and technological innovation, and further drive the evolution of social innovation form [3].

Advanced concepts such as “digital indigenous people,” “Internet +,” “smart education,” “maker education,” and “core literacy” are constantly changing people's minds. For these changes, China has implemented the “Primary and Secondary School Teachers Training Projects,” “Modern Distance Education Project of Rural Elementary and Middle Schools,” “Three Links and Two Platforms Construction,” and other series of education informatization strategic projects. But the integration between modern information technology and education is far behind the other industries. The situation of rural areas and underdeveloped areas is not optimistic. “Integration” has become a “high-frequency word” in the policies and guidelines of educational institutions at all levels and a hot topic for researchers and practitioners [4]. With the confusion of the above problems, the classroom development mode of higher-order thinking supported by technology as the research topic was chosen to enrich the influence of environment on the development of higher-order thinking and its rules through technology. The general theoretical and practical model was explored, which provided theoretical, practical, and methodological perspectives for the research on the development evaluation of higher-order thinking, development strategies, cognitive diagnosis, and teaching intervention. More importantly, it was expected to trigger some thoughts on the improvement and better development of the integration of educational informatization and technology. Therefore, the relationship between technology and thinking development was the starting point of the research. Technology-enriched environmental features and interpretation of higher-order thinking ontology were the bases of the research. The core task of the research was to enrich the influence of the classroom environment on the development and change of higher-order thinking, and how to build an operable higher-order thinking development model [5]. The specific problems are sorted out, as shown in Figure 1.

What is the status quo of the cultivation and development of higher-order thinking? What factors and conditions is it affected by? It is found that higher-order thinking began to attract attention from 2008 and then it has been on the rise. Through the research on the cultivation mode, development conditions, supporting environment, and influencing factors of higher-order thinking, it is found that the research categories and perspectives are diverse [6]. The research categories and perspectives are diverse and unfocused. It is mainly based on the research of a certain technology or a certain discipline with higher-order thinking goals. From the technical perspective, it mainly focuses on information technology, network environment, and digital resources, which can be specifically divided into social software, semantic web, Wenqest, gamification teaching, flipped classroom, etc. From the theoretical perspective, it includes constructivism, cognitive apprenticeship, deep learning, and so on. From the perspective of teaching and learning activities, it includes teaching design, digital environment design, learning mode, teaching strategy, teaching mode, and so on. Learning methods include problem solving, exploration, research, etc. High frequency words are technology and its role, thinking environment, resource type, learning mode, learning behavior, teaching mode, teaching behavior, teacher knowledge, student experience, teaching problem-solving strategies, and so on [7]. Among them, the difference between high-order thinking and low-order thinking is shown in Figure 2.

It is guided by high-order teaching objectives and driven by real problems or tasks, which focuses on meaningful learning and integration with specific teaching. Information technology is as a learning tool and intelligent partner of learners. It creates learner-centered learning environment and changes the roles of teachers and learners. It creates an ideal interactive environment to promote development through evaluation. It also provides a theoretical framework for the teaching design of higher-order thinking by means of semantic composition of target, learning task, teacher role, information technology role, learning evaluation, and learner role in the whole hypothesis model [8], as shown in Figure 3.

## 2. New Media Concept and Basic Theory

Advertising image is one of the basic elements of information construction and plays a particularly important role in advertising information dissemination. However, in the new era of social culture and intelligent technology integration, advertising forms are also evolving, including the new connotation of advertising language, namely, language image. In the era of new media, it is more and more difficult for single and static advertising to ensure the effectiveness of advertising information transmission, while advertising design completed through multi-dimensional, virtual reality, media interaction, and other ways is more and more popular. Advertising information achieves the two-way transmission and the connotation of advertising is also evolving [9]. A series of artistic design rules such as rhythm, balance, contrast, and unity are used to better express the sense of form and beauty of advertising. This can be called the language of advertising. Images in the new media era focus on “communication,” that is, two-way interaction, which requires the further expansion of comprehensive sensory and thinking cognition of the target groups. See Table 1.

The connotation of new media advertising language image and image is constantly expanded and extended in the interaction of environment, until dynamic, until apperception sharing. It shows different degrees of stereoscopic deepening and mutual integration both horizontally and vertically. In a sense, the language image can also be a kind of image. And the image can also be continuously expanded and extended in the interaction of a kind of context until it becomes dynamic and even apperception sharing [10]. Horizontally and vertically, it shows different degrees of stereoscopic deepening and mutual integration. In a sense, language image can also be a kind of image and image can also be a kind of language image. The two gradually move from disjoint parallel relationship to symbiosis, as shown in Figure 4.

In the research, apperception sharing mainly refers to how the language image elements and the audience's perceptual experience are skillfully combined to achieve harmony and unity in new media advertising. The relationship between language image and apperception sharing is a two-way interaction. The combination of language image and image provides the medium and form for the realization of apperception sharing. Conversely, the realization of apperception sharing further provides feedback for new media advertising. As shown in Figure 5, the two-way interaction between the two is further towards “integration” [11].

For the focus of new media advertising research, language symbols can convey the meaning of advertising content. The advertising language symbol is located in the middle layer. The innermost layer is the representation of the advertising content and the outer layer is the perception and interaction of the advertising audience. It can be called “concentric circle” relation in new media advertisement. As shown in Figure 6, it is the semiotic basis to further explore the relationship between them [12].

When language symbols are used in new media advertising, the connotation of advertising language symbols also deepens between language symbols and advertising images, and its connotation even goes beyond the description of advertising images. The mutual contradiction is also the basis and condition of the interaction between language image and image to realize “sharing,” as shown in Figure 7 [13].

Due to the understanding of the human brain and the subjective active role in understanding objective things, it has a certain degree of masking and concealment. Its deep meaning is often not easy to detect, so we often only see some visual illusions to believe in it. The image of new media advertisement has the division of connotation layer and epitaxial layer. In addition to the surface information, there is also the deep meaning of mixed information. Its structure is shown in Figure 8.

In addition, the transmission of new media advertising information is based on “common experience.” It relies on the shared experience between the advertising designer and the advertising recipient group, and eventually forms the intersection set of brain ideas, contributing to what we call the new media advertising symbols with conventional characteristics, as shown in Figure 9.

## 3. Research on Learning Adaptability of Technology Support

### 3.1. The Generation Mechanism of the Internal Meaning of Language Image and Image

After the language image in the new media advertisement enters the human brain, it will also produce the corresponding image, which is a kind of reconstruction imagination. Taking the new media advertising as a whole, the whole will be like a mirror [14]. There is a similar refraction of life, and these refractions are from people's prior feelings to adapt to this. Images in new media advertisements or the audience's first impression of the target object project corresponding concepts in their minds, and eventually transform into language symbols. See Figure 10.

The language image and image in new media advertisement are two parallel and disjoint “paraphrase chains.” However, they can generate new connotations through the interaction of language diagrams and extend countless interactive paraphrase chains. Just like Pierce's triangle relationship, the intricate relationship between multiple images and images generates a complex “network” of new media advertising meanings, which can loop and extend indefinitely [15].

In new media advertising, the tension between the language image and the image fluctuates around the form and effectiveness of the advertisement, which is generally positively correlated. When the tension of the language image increases, the effectiveness of the advertisement also increases [16]. Similarly, when users' multi-senses participate in the cognition of objective things, there is a linear relationship between the effectiveness of advertising and the realization of “apperception sharing.” The higher the effectiveness of advertising, the greater the realization of apperception sharing. See Figure 11.

Secondly, multi-sensory participation helps to maximize the effectiveness of advertising. Taking the above materials as the research object, combined with the secondary data of relevant studies, it is concluded that the stimulation and influence of single sensory participation and multi-sensory participation on people's psychology are different. See Table 2. Data show that advertisements with multi-sensory participation have better effects on the psychological and behavioral aspects of target groups than advertisements with single sensory participation. The standard deviation value proves that rich sensory participation can effectively reduce the deviation degree of people's cognition of advertising information [17].

### 3.2. The Research Overview of Learning Adaptability of Technology Support Abroad

#### 3.2.1. Time Span Analysis

In the research, the total literature of technology-supported learning adaptability, technology-improved learning adaptability, and technology-environment learning adaptability were analyzed [18]. Among them, the literature on learning adaptability in the technical environment could be further divided into the literature on learning adaptability in the hybrid learning environment and the literature on learning adaptability in the network learning environment, as shown in Figure 12.

At present, the research on the learning adaptability of technology support in China only includes the research on the learning adaptability under the technology environment (hybrid learning environment and network learning environment). In addition, there are few researches on learning adaptability in mixed learning environment [19]. Therefore, this article combines researches on learning adaptability in network learning environment and hybrid learning environment for analysis, and obtains the time span of research on learning adaptability of technology support at home, as shown in Figure 13.

This article systematically summarizes the research situation of hybrid learning at home and abroad and the research status of the learning adaptability of technology support, obtaining valuable enlightenment and laying a foundation for the follow-up research. Through the summary, specific Revelations are as follows [20]:

1. Research on hybrid learning at home and abroad presents two important trends. Specifically, the first one is to further study the teaching and learning rules in the hybrid learning environment and to explore new hybrid learning methods, such as MOOC-based hybrid learning. Through in-depth exploration of its teaching and learning rules, teaching activities or modes are designed to improve teaching quality and promote the reform of higher education today [21]. The second one is that the research perspective gradually turns to the micro level exploration, focusing on how students learn and how to promote students to learn effectively. Among them, learning psychology is an important research topic in the current hybrid learning, mainly involving the psychological characteristics and laws of students in the hybrid learning environment, including learning attitude, learning emotion, cognitive and metacognitive laws, learning motivation and self-efficacy, etc. Learning adaptability, as a hot research topic in the field of learning psychology, emphasizes the positive adjustment of students' inner psychology and external behavior, which covers many psychological and behavioral elements in the learning process.
2. More and more scholars are paying attention to the research of the learning adaptability of technology support. In terms of the research overview of learning adaptability (time distribution, major journals, and important literature), it can be seen that the research on learning adaptability under technology-supported environment began in 1999 and 2004, respectively. The research on the learning adaptability of technology support in China began in 2002 and the research on the learning adaptability of hybrid learning environment began in 2015. The development of foreign research is earlier than domestic research. The overall number of research is also more than that of domestic research. The research system is relatively more mature. In addition, in terms of research trend, the number of literature both at home and abroad is on the rise, which also indicates that more and more scholars begin to pay attention to the research of the learning adaptability of technology support.
3. The research of the learning adaptability of technology support includes a wealth of topics. This part mainly expounds the research of learning adaptability under technological environment and the research of technology improving learning adaptability. Firstly, the research of learning adaptability in technological environment, including hybrid learning environment and network learning environment. Through a detailed review of domestic and foreign literature, it is found that there are relatively few researches on learning adaptability in hybrid learning environment at present, which mainly include four topics, namely, research on the status level and countermeasures of learning adaptability, research on influencing factors of learning adaptability, research on the correlation of learning adaptability and research on the intervention of learning adaptability [22].

## 4. Research on the Development of Higher-Order Thinking and Causal Structure Effect

### 4.1. Thinking Structure ESEM Exploratory Structure Analysis

#### 4.1.1. Research Methods and Survey

Since the potential relationship structure between observation variables and factors of the designed higher-order thinking structure was not clear in the previous researches, the research adopted the factor analysis method commonly used in capacity structure to reduce the dimensionality of the obtained data and then established the higher-order thinking structure factor model on the basis of determining the potential common factors. In the process of specific research, the SPSS tool was first used to explore the functional advantages of factors. The factor analysis method was used to find common factors between latent variables to achieve the purpose of dimensionality reduction and structure simplification and the preliminary common factor type was obtained. However, this method was subjective and lacked the test of fitting actual data and theoretical model. Therefore, exploratory structural equation modeling (ESEM) was used to explore the factor structure of higher-order thinking flexibly and verify the function and advantage of its factor model systematically, so as to provide a more suitable measurement model for the analysis of the relationship between the latent variables of higher-order thinking structure. In the process of specific factor analysis and extraction, considering the complexity and overall characteristics of higher-order thinking structure as well as the correlation between various factors, the maximum fitting method was chosen, which could generate correlation matrix in the process of factor extraction. For factor rotation, Promax (also known as optimal skew method) was adopted in the skew axis method, which made the previous relationship of factors well represented and overcame the disadvantage of direct method that the assumed factors were independent and unrelated. In the investigation, a large sample survey and sample test were adopted, which met the requirement of maximum fitting method and skew rotation that samples were more than 200 and normally distributed.

On the basis of field lectures and interviews, stratified random sampling method was adopted in the research. And questionnaires were distributed at four levels, including developed regions, moderately developed cities, county-level cities, and towns. In the process of questionnaire distribution, the method of filling in and collecting the questionnaire in the classroom was adopted. A total of 1565 questionnaires were collected, of which 1505 were valid. The total samples were randomly divided into two types of independent samples, among which 656 samples were subjected to exploratory factor analysis. Male and female students accounted for 44.97% and 55.03% of the questionnaire, respectively. Another 849 samples were analyzed for ESEM and confirmatory factor analysis. Male and female students accounted for 48.4% and 50.5% of the questionnaire, respectively, and the missing value accounted for 1.1%. The male-female ratio, grade, and regional distribution of the two independent samples were basically balanced.

#### 4.1.2. Normal Distribution Test

Normal distribution is the basis of many tests, such as the *F* test, *t* test, chi-square test, etc. The independent sample *t* test and one-way ANOVA used in the research are the *t* test and *F* test used. Therefore, it is necessary to test the sample distribution. Sample normality test methods include graphic method, skewness kurtosis test method, and nonparametric test method.

P-P graph, Q-Q graph, and histogram are commonly used in the graphical method, among which the Q-Q graph is more efficient. The Q-Q diagram takes the quantile of the sample as the abscissa, the corresponding points calculated according to the normal distribution as the ordinate, and the sample representation as the scatter point of the cartesian coordinate system. If the data follow a normal distribution, the sample points should be distributed diagonally around the first quadrant.

In the skewness kurtosis test, sample skewness coefficient is *S*=*B*_3_/(*B*_3_)^3/2^, which is used to test symmetry. When *S* > 0, the distribution is positively skewed. When *S* < 0, the distribution is negatively skewed. Sample kurtosis coefficient is *K*=*B*_3_/(*B*_3_)^2^ − 3, which is used to test the kurtosis. *K* > 0 is the peak distribution. *S* < 0 is flat distribution. When *S* = 0, *K* = 0, it is normal distribution. In normal distribution, skewness coefficient and kurtosis coefficient are close to 0. If *S* > 3 and *K* > 8, researchers need to start paying attention. If *K* exceeds 20, researchers need to pay close attention.

Nonparametric test is a method to use sample data to infer the pattern of population distribution when the population variance is unknown or little known. The nonparametric test method is named “nonparametric” test because it does not involve parameters related to the population distribution in the inference process. Nonparametric test methods are commonly used *W* test, goodness of fit test, etc. In the research, skewness kurtosis test was used to test the normality of samples. Most of the absolute values of skewness coefficient and kurtosis coefficient of the samples in the research were less than 1 and very few were less than 2, indicating that the skewness coefficient and kurtosis coefficient were significant. Therefore, the sample of the research basically conformed to the normal distribution. In the research, the skewness coefficient and kurtosis coefficient of the grouped samples involved in the independent sample *T* test and one-way ANOVA were also calculated by SPSS, both of which were significant.

### 4.2. Investigation on the Status Quo and Application Potential of Technology-Enriched Classroom Environment

In the part of the survey, the method of random stratification was adopted. The six regions to be investigated were stratified according to their economic development level and educational development level and samples were randomly distributed to schools selected at each level. A total of 880 questionnaires were collected, of which 849 were valid, with an effective rate of 94.67%. The proportion of boys and girls was 48.4% and 50.5%, and the missing value accounted for 1.1%. The technical environment survey of the school found that the technical facilities of the school were more concentrated in the construction of multimedia classroom, computer classroom, and campus website, accounting for 28.0%, 27.2%, and 17.7%, respectively.

### 4.3. Application Potential Analysis

Based on the overall investigation and comparison of the status quo of technology-supported learning environment, the following conclusions and reflections can be drawn based on the potential of students to adapt to technology-enriched learning environment.

1. Emerging technologies such as social media promote interactive and rich learning environments. The development of new technology has promoted students' choice of technology. Due to the instantaneity and interactive characteristics of emerging technologies, Wechat and public accounts are sought after by classes, students, and teachers, have and become the most used communication tools among students and teachers. However, the application of QQ and class QQ group has been gradually weakened, and teachers, students, and classes have entered the stage of social media.
2. Personalized learning and teaching space has become a new feature of technology application. The application of micro-blog, personal website or space, Wechat public account, and other technologies has been widely concerned in classes, teachers, and students. Personalized learning and teaching and the establishment of their own personal learning and teaching space are the current trend of technology application that teachers and students are concerned about and enthusiastic about.
3. Learning based on integrated resources such as electronic schoolbags has become a new development trend. Electronic backpacks or resource packs have become a hot topic of concern for classes, students, and teachers, especially senior students. The interaction, integration, personalization, learning analysis, and evaluation functions of e-book packages can better promote students' learning, and teachers and students pay more and more attention to them. In addition, with the development of virtual technology and simulation technology, virtual technology began to be concerned in some developed areas, and students began to adapt to and accept the classroom virtual situational teaching.

In conclusion, the integrated attention and application of technology by schools, classes, students, and teachers will promote the application of technology in the classroom environment. The change of educational information construction and concept in schools and the promotion of some experimental projects will also stimulate the construction and investment of technology-enriched classroom environment in schools, and stimulate the potential application of technology by classes, teachers, and students, so as to form a good technology-rich classroom environment atmosphere. The research is innovative in theory, method, and practice. The research results provide a new perspective for higher-order thinking teaching and evaluation under the background of education informatization, and provide a good practical model for optimizing digital resources and environment, and improving students' cognitive level and skill diagnosis, cognitive strategy optimization, and precision teaching intervention. The practical application and improvement of the model will also be the focus of further research.

## 5. Conclusions

The continuous development of intelligent technology has greatly enriched the information transmission form of new media advertising. In the research, the “newness” of new media advertising was taken as its base, the relationship between language and image in advertising was re-examined, and the internal mechanism of realizing “apperception sharing” in new media advertising was summarized. It not only enriched the relevant theory of advertising language graph relationship but also provided certain reference and guidance for the design practice of new media advertising to some extent. And the development of advertising in the era of new media is changing with each passing day, showing a spiral trend. Tomorrow's new media will no longer be the phenomenon we are familiar with today. The connotation of language image and image will be more and more dynamic and situational, and the boundary between each other is gradually melting. People's sensory function is no longer mainly audio-visual. Multidimensional sensory channels are mobilized and integrated. The overall role of apperception is becoming more and more obvious. Under the support of advanced media technology, unique presentation form, and comprehensive feedback of people's multiple senses, new media advertising gradually realizes “apperception sharing,” which also proves the practical significance of the research.

But because of the limited time and energy, there are still a lot of deficiencies to be improved. For example, in advertising design, not all things can use the data to measure and analyze. The change of people's emotion tends to be very subtle, which is not quantitative. But the research advertising still plays a guiding role in the development of new media. The development of new media is rapid, but the overall research on it is still at a relatively shallow level. The “apperception sharing” of new media advertising needs to be promoted by a large number of practices, and the deep value of language and image also needs to be continuously explored by relevant scholars. The research is expected to provide a beneficial attempt for the research of new media advertising.

## Figures and Tables

**Figure 1:** Presenting the problems.

**Figure 2:** High-order thinking and low-order thinking.

**Figure 3:** Hypothesis model of thinking teaching design.

**Figure 4:** The extension and expansion of the connotation of language image and image.

**Figure 5:** Language graph relationship and apperception sharing.

**Figure 6:** Diagram of concentric circle relationship in advertisement.

**Figure 7:** New media advertising language image.

**Figure 8:** New media advertising image from the perspective of semiotics.

**Figure 9:** Diffusion of shared experience.

**Figure 10:** Symbol chain of language graph transformation.

**Figure 11:** Relationship between new media advertising effectiveness and “apperception sharing.”

**Figure 12:** Time distribution of research on learning adaptability of technology support abroad.

**Figure 13:** Time distribution of research on learning adaptability of technology support at home.

**Table 1:** Changes of connotation of advertising language image.

Advertising image	Form	Content	Characteristics	Summary
Traditional advertising image	It has a fixed form. It is attached to a specific medium	Advertising language, text, etc., to explain advertising information	Two-dimensional, unidirectional, stationary	Advertising language and social conventions commonly known as word signs
New media advertising image	There is no fixed form. Digitize. Advertising information is displayed in the form of digitization	Communication elements and forms of advertising information	Three-dimensional, two-way interaction, apperception sharing	All media and means used to perceive, communicate, communicate, , and deliver advertising information

**Table 2:** Comparison of single sense and multi-sense.

	Single sense		Two senses		Three senses	
	Average	Standard deviation	Average	Standard deviation	Average	Standard deviation
Cognition	1.79	0.893	2.39	0.527	3.20	0.483
Mood	1.70	0.810	2.23	0.726	2.36	0.695
Attitude	1.52	0.755	2.09	0.663	3.26	0.645
Memory	1.55	0.617	2.12	0.432	2.55	0.357
Action	1.79	0.927	2.24	0.812	2.29	0.655

## Data Availability

The labeled data set used to support the findings of this study is available from the corresponding author upon request.
